# The Effect of Acceptance and Commitment Therapy on Psychological Nursing of Acute Cerebral Infarction with Insomnia, Anxiety, and Depression

**DOI:** 10.1155/2022/8538656

**Published:** 2022-06-22

**Authors:** Xinyu Wang, Jie Chen, Yun-e Liu, Yan Wu

**Affiliations:** ^1^Department of Outpatient, PLA Rocket Force Characteristic Medical Center, Beijing 100088, China; ^2^Department of Vascular Neurosurgery, PLA Rocket Force Characteristic Medical Center, Beijing 100088, China; ^3^Department of Neurology, PLA Rocket Force Characteristic Medical Center, Beijing 100088, China

## Abstract

Acute cerebral infarction (ACI) is a kind of stoke, mostly suffering from insomnia, anxiety, and depression; therefore, the importance of psychological nursing in such patients is a necessary mean. Acceptance and commitment therapy (ACT) is a psychological theory which advocates embracing pain, improving the ability to face pain, with the goal of improving psychological flexibility, so as to reduce the negative impact of pain on personal life. To explore the effect of psychological nursing intervention on ACI patients with anxiety, depression and insomnia are based on acceptance and commitment therapy. A randomized clinical trial study was conducted on 140 eligible ACI patients suffering from insomnia, anxiety, and depression who were selected using easy sampling methods and allocated randomly into two groups of observation and control. The data were collect through demographic questionnaires, the summary of Pittsburgh sleep quality index (PSQI), Athens Insomnia Scale (AIS), Acceptance and Action Questionnaire-II (AAQ-II), Cognitive Fusion Questionnaires (CFQ), Self-Rating Depression Scale (SDS), and Self-Rating Anxiety Scale (SAS). The observation group received ACT treatment, while the control group received standard care. The scores of AAQ-II and CFQ were significantly decreased in the observation group, indicating that psychological flexibility was improved (*P* < 0.05); the scores of SAS and SDS were significantly decreased in the observation group; and the scores of PSQI and AIS were significantly decreased in the observation group. The difference between the two groups was verified by *t*-test.

## 1. Introduction

Acute cerebral infarction (ACI) is a cerebrovascular disease with complex pathogenesis [1]. ACI patients are prone to insomnia under the action of multiple factors, leading to poor sleep quality and even secondary ACI [2]. Studies have shown that up to 56% of ACI patients suffer from insomnia [3]. ACI patients with anxiety, depression, emotional imbalance, anger tendency, etc., unable to contact with the status quo or achieve the target and value, namely, psychological flexibility was decreased. They lack the ability to adjust their negative emotions, cannot accept the status quo, correctly understand the significance of rehabilitation training, and resistance to the status quo or unable to do anything about the ambivalence; this psychological state is inflexibility. Thus, it causes a series of psychological problems such as ineffective denial, adjustment disorder, self-image disorder, anxiety, and mental distress. These psychological problems will lead to insomnia, reduced sleep quality, and affect the prognosis of patients. However, the severity of these psychological problems is far from anxiety, depression, and other aspects of psychiatric diagnosis, but requiring nursing staff to implement psychological nursing. Acceptance and Commitment Therapy (ACT) [4] advocates embracing pain and improving the ability to face pain, aiming at improving psychological flexibility, so as to reduce the negative impact of pain on personal life. The ACT theory includes 6 parts: flexible attention to the present moment, acceptance, cognitive defusion, self-as-context, committed action, and valuing. Many studies [5–11] have applied it to the psychological care of patients and their families, such as relieving the fear of patients with recurrent oral cancer, improving the self-management ability of patients with chronic diseases, alleviating the mental health problems of the population such as maternal depression after painless delivery, or improving the self-management ability of patients with diabetes.

An 8-week ACT therapy course decreased stress and other psychological health indices in people with IBD in a randomized controlled experiment. They have all had a positive psychological nursing effect in a short amount of time, namely, during their hospital stay, and they have all focused on enhancing psychological flexibility, improving sleep and other health issues, and boosting patients' quality of life. ACT has been found in studies to enhance not only physical function but also a variety of mental health issues [12]. Many studies at home and abroad have shown that psychological flexibility reflects mental health level to some extent [13]. However, we found no studies that applied this model to ACI patients such as those with insomnia, anxiety, and depression. Therefore, the present study aims to examine the effects of interventions according to ACT on psychological nursing.

The following is a summary of the research: Section 2 contains the patients and methods.  Section 3 discusses the results and experiments.  Section 4 consists of the discussion section; finally, the conclusion brings the paper to a finish in Section 5.

## 2. Patients and Methods

### 2.1. Trial Design and Participants

This study was a randomized clinical trial. 100 patients were enrolled in the study including 50 patients for the observation group and 50 patients for the control one. Two groups of patients were selected and randomly assigned to observation and control groups. Patients in the observation group received psychological nursing which based on ACT and were carried out according to the nursing steps of assessment, diagnosis, planning, implementation, and evaluation; patients in control group received traditional psychological nursing which included assessment, comfort, communication, and music therapy. Observation group comprised 39 cases of male and 11 cases of female, with an average age of 62.04 years old. Control group consisted of 38 cases of male and 12 cases of female, with an average age of 60.86 years old, and the self-care model components in the two groups were compared using independent samples *t*-test or Chi-squared test. As revealed, no significant difference was evident prior to intervention in terms of gender (*P* = 0.812) and age (*P* = 0.798). Anxiety, depression, insomnia, and psychological flexibility were compared between the two groups before and after 1 month of psychological nursing.

### 2.2. Selection Criteria

The inclusion criteria were as follows: (1) over 18 under 75 years of age, (2) the vital signs were stable, (3) be able to communicate face to face normally, (4) PSQI ≥ 11 points and AIS ≥ 6 points, (5) SAS ≥ 49 points, and SDS ≥ 53 points. Exclusion criteria consisted (1) previous history of mental illness (such as bipolar disorder) or dementia, history of use of psychiatric drugs or sedatives within 6 months, or use of antidepressants and other drugs; (2) transient cerebral ischemia patients; (3) severe anxiety and depression (SAS ≥ 69, SDS ≥ 73); (4) a history of substance abuse or dependence; (5) psychotherapy in the past 3 months.

### 2.3. Data Collection and Statistical Analysis

#### 2.3.1. Data Collection Tools

1. *PSQI*. The scale [14] can be used to assess sleep quality in patients with sleep disorders and mental disorders, as well as in typical persons; the total score ranges from 0 to 21, with higher scores indicating poorer sleep quality
2. *AIS*. There are 8 items in this scale [15], and each item can be divided into four grades from none to severe: 0, 1, 2, and 3. And the total score is less than 4: no sleep disorder; if the total score is 6: suspicious insomnia; if the total score is above 6: insomnia. The main content of this scale is the subjective feeling of sleep
3. *SAS*. The scale contains 20 items [16] to reflect the subjective feelings of anxiety and adopts 4-level scoring. Reverse scoring is required for the 5th, 9th, 13th, 17th, and 19th; and normal scoring is required for the rest. The total score of 20 items is rough, which is multiplied by 1.25 for standard score. The standard score is based on a cutoff of 50, a score below 49 is normal, a score between 50 and 59 is mild anxiety, a score between 60 and 69 is moderate anxiety, and a score above 69 is severe anxiety
4. *SDS*. This scale was compiled in 1965 and contains 20 items to reflect subjective feelings of depression [17]. It adopts a 4-level score, among which 10 items need reverse score and the rest are normal score. The total score of 20 items is rough score, which is multiplied by 1.25 for standard score. The cutoff score was 53, with a score below 53 considered normal, 53-62 considered mild depression, 63-72 considered moderate depression, and 73 or above considered major depression
5. *AAQ-II*. The questionnaire is designed to assess the degree of “empirical avoidance.” There are seven items on the scale, ranging from 1 (never) to 7 (always). The higher the score, the more empirical avoidance is present. “Empirical avoidance” [18] is an act that people attempts to change the form, frequency, or sensitivity of their internal experiences (such as thoughts, emotions, and somatosensory sensations) in their minds, even if doing it can lead to actions that are inconsistent with their personal values or goals (such as giving up pursuing a long-term goal in order to avoiding anxiety)
6. *CFQ*. “Cognitive Fusion” is the tendency of people's behavior to be excessively controlled by language rules and thought content, which will enable individuals to automatically extract the literal meaning of thought events, and thus unable to guide their behavior with the direct experience of the “here and now” [19]. There are 9 items in the scale [20], with points from 1 (never) to 7 (always), the score higher, the degree deeper of cognitive fusion

#### 2.3.2. Statistical Analysis

Double entry for verification data, SPSS 22.0 was used for data analysis, and the data was checked by statistical experts. The measurement data is described by the mean ± standard deviation (SD). And the enumeration data is described by frequency and composition ratio. *T*-test and nonparametric tests were used for measurement data, and chi-squared test was used for enumeration data. *P* < 0.05 was considered as significant difference.

### 2.4. Intervention Measures in Observation Group

#### 2.4.1. Psychological Nursing Assessment

Psychological flexibility, anxiety, depression, and insomnia were evaluated with the scale before intervention. There was no significant difference in scores between the two groups, as shown in Table 1. Patients were closely observed and communicated frequently to find out their negative emotions, and some common negative statements and body language were recorded for psychological nursing evaluation to facilitate diagnosis.

#### 2.4.2. Psychological Nursing Diagnosis

In combination with the psychological nursing evaluation content and clinical commonly used psychological nursing diagnosis, PES structure is used to carry out psychological nursing diagnosis, and generalized diagnosis of patients is summarized, as shown in Table 2. The psychological nursing diagnosis of PES structure corresponded to the contents of psychological nursing evaluation and the six problems of psychological flexibility, and the various symptoms or signs in the psychological nursing diagnosis of PES structure belonged to the symptoms of psychological inflexibility. The details are shown in Table 3.

The “symptoms” in Table 3 are compared with those in Table 2. For example, “P-① -S-c” is the “symptom- c(Willfully ignoring certain symptoms and dangers)” in “item S” corresponding to “① invalid denial” of “item P” in Table 2.

#### 2.4.3. Planning and Implementation

According to the basic concept of the psychological nursing plan, this study's psychological plan includes the following: ACT psychological nursing diagnosis, predicted goals, psychological nursing measures, and evaluation,

1. *Nursing Diagnosis*. The patient's ACT psychological nursing diagnosis is summarized according to the results of the assessment and diagnosis. The reduced psychological flexibility leads to anxiety, depression, and insomnia
2. *Expected Goals and Measures*. According to ACT, psychological nursing measures are formulated and divided into 7 units, as shown in Table 4

## 3. Results

The comparison of the results of the two groups 1 month after intervention is also the evaluation process of psychological nursing. Compared with before intervention, the scores of both groups are improved, but the observation group is significantly better than the control group, as shown in Table 5.

## 4. Discussion

There were 6 psychological nursing diagnoses in this study, and after removing the overlapping etiology, there were still 20 etiologies (E) and 21 symptoms (S). However, when ACT was diagnosed with psychological nursing for patients, there were only one problem of reduced psychological flexibility, and there were 6 manifestations of low psychological flexibility. Patients suffered from experience avoidance, cognitive fusion, and psychological inflexibility, according to the findings of this study. Acceptance and action refer to the patient's desire to feel their feelings and move on from those undesirable psychological experiences. Acceptance and action in this study refer to patients' acknowledgment of their sickness, as well as their negative emotions and symptoms following the illness. In this situation, they can still have a good living state and beliefs in a worse living environment than before the illness.

In this study, ACI patients often held a pessimistic attitude towards the prognosis of the disease, believing that the disease was worthless because of the inconvenience of movement after the disease. Because ACI is a chronic disease with a high disability rate, many middle-aged and elderly people will change their roles and reduce their adaptability, which causes its occurrence anxiety depression and causes insomnia. By contrast, ACT makes psycho-care diagnosis simpler, attributes all symptoms to a single problem of “reduced mental mobility,” and develops a more comprehensive program that starts with six signs of low mental mobility.

If a mental care program is developed based on the diagnosis of psychological care for 6 health problems (P), 21 symptoms (S) resulting from 20 causes (E) need to be addressed, involving more psychological techniques and psychological nursing techniques. Make the plan long and complicated, without a full set of scientific theory support. And ACT is only to counter the problem of psychological flexibility, improve psychological flexibility, not committed to solve the symptoms, but has the abilities such as acceptance of the status quo, let patients see negative thoughts in the mind of the border, better aware of the current situation, in this kind of situation, has the ability to face the pain, solve the symptoms that are caused by negative emotions, to relieve negative emotions and improve clinical purpose of adverse symptoms. A great number of research have indicated that strengthening patients' psychological flexibility is critical to resolving the symptoms of psychological issues. The use of ACT in the development of a psychological nursing plan so that patients take the initiative to accept negative emotions and problems, and in this situation, to find their own value direction and put it into action in order to alleviate negative emotions, improve insomnia, and improve their quality of life. Higher psychological flexibility enables patients to face life more positively in painful situations and reduces the generation of negative emotions and the impact of negative emotions. Studies have shown that psychological flexibility reflects mental health.

ACT is a professional psychological technique with scientific theoretical basis and a complete practical process to support its use in psychological nursing. This study standardized the process of psychological nursing, diagnosed patients with common problems, and preliminarily constructed a more professional and detailed program, and the application effect is good, and patients' psychological flexibility can be improved, relieve anxiety and depression, and improve insomnia symptoms. However, in the specific implementation, there are still some personalized problems. More attention should be paid to patients' psychological flexibility, more care should be given to patients, social support should be strengthened, value direction should be found in the hardship, and action should be taken to lead a positive and optimistic life in order to train medical staff to learn ACT. However, this study was only initially applied in ACI patients, and the acceptance of ACT psychological nursing among patients of different ages should be further explored to develop a scale to measure the psychological flexibility of sACI patients for a more detailed and accurate measurement. And explore the psychological nursing effect of the best nursing frequency, in order to clinical work for reference.

## 5. Conclusion

In general, using ACT in psychological nursing can help ACI patients improve their mental flexibility, decrease negative emotions like anxiety and depression, and improve insomnia symptoms, sleep quality, and overall quality of life. At the same time, the process and scientific basis of psychological nursing plan formulation are explained. This study is innovative and reproducible and has certain clinical significance. And “ACT ⟶ psychological nursing ⟶ psychological flexibility ⟶ relief of negative emotions ⟶ improvement of adverse symptoms” can be used as a new way to explore psychological nursing.

## Figures and Tables

**Table 1:** Comparison of scales before psychological nursing.

Item	Scores (min-max)		*Z*	*P* value
	Observation group	Control group		
SAS	61.00 (60-66)	61.50 (60-66)	-0.240	0.811
SDS	67.50 (62-72)	67.00 (63-72)	-0.021	0.983
PSQI	15.00 (11-19)	14.00 (11-18)	-1.139	0.255
AIS	13.00 (8-17)	12.00 (8-17)	-1.439	0.150
AAQ-II	40.00 (34-47)	39.00 (34-47)	-1.087	0.277
CFQ	55.00 (45-64)	54.50 (45-64)	-0.674	0.500

**Table 2:** Psychological nursing diagnosis for patients.

P (problem)	E (etiology)	S (signs and symptoms)
(1) Invalid denied	(a) Relating to the generation of denial of a particular scene (b) Associated with the observed overstimulation of the disease (c) Associated with ACI	(a) Delay or refuse rehabilitation training (b) Refusing to talk about the pain caused by the disease, and making gestures or remarks of dismissal when talking about painful things (c) Willfully ignoring certain symptoms and dangers
(2) Impaired adjustment	(a) Associated with impaired physical mobility after ACI that causes changes in lifestyle (b) Associated with damage to self-esteem (c) Related to insufficient support systems	(a) Self-reported inability to accept changes in health status (b) Too long denial of changes in health status, showing anger (c) Lack of practical action to solve the problem and future-oriented requirements
(3) Self-image disorder	(a) Associated with ACI (b) Related to mental stress from social environment (c) Conflicts with others' acceptance of human appearance (d) Related to patients' expectations of appearance and activity requirements	(a) Negative responses to existing changes in bodily function, feelings of shame, guilt, and disgust (b) Avoid talking about the function of altered parts of the body (c) Have pain, depression, sadness, and other negative emotions (d) Avoid social contact
(4) Presentimental sadness	(a) Relating to the loss of work capacity and social status (b) Relating to the prospect of loss of property (c) Relating to the lack of effective support (d) Associated with a lack of experience in dealing with ACI (e) Associated with ACI	(a) The patient has a premonition that important things will be lost and shows negative emotions about the expected loss (b) Withdrawal behavior, loss of interest in life, changes in daily activities, and ambivalence (c) Excessive emotional reaction, denial, self-blame, depression, anger, and anxiety (d) Changes in physiological function and sleep disorders
(5) Spiritual distress	(a) Associated with life-threatening (b) Related to the loss of some self-care ability and social status (c) The value of fuzzy	(a) Abnormal behavior and emotions, crying, withdrawal, anxiety, depression, anger, and denial (b) Significant changes in sleep and mental outlook (c) Express doubts about their own values and thus feel spiritually empty (d) Seek spiritual sustenance and spiritual help
(6) Anxiety	(a) Relating to a premonition that the patient's health is at risk (b) Associated with threats to self-concept (c) Associated with a premonition of misfortune	(a) Abnormal emotions and behaviors such as speaking too fast, helplessness, and self-accusation (b) Too much attention to oneself and self-reported worries and worries (c) Inability to concentrate, repeat aimless movements, and avoid behavior

**Table 3:** Psychological inflexibility problems for patients.

Psychological inflexibility	Symptoms	Emotional symptoms	Physical symptoms
Cognitive fusion	P-①-S-c,P-④-S-a	Moderate anxiety Moderate depression P-③-S-c P-④-S-c P-⑤-S-a	Insomnia P-④-S-d P-⑤-S-b
Experiential avoidance	P-①-S-b,P-③-S-bd, P-⑤-S-a,P-⑥-S-a		
Self-as-content	P-③-S-a,P-⑥-S-b		
Inflexible attention	P-②-S-ab,P-④-S-a		
Lack of contact with chosen values	P-④-S-b,P-⑤-S-cd,P-⑥-S-c		
Avoidant persistence	P-①-S-a,P-②-S-c		

**Table 4:** ACT psychological nursing measures.

Times	Unit content
No. 1	Get of your mind, understand ACI
Basis: ACT—cognitive defusion	
Location: ward; time: after the end of basic treatment in the morning; supplies: knowledge album, mobile phone.	
(1) Encourage patients to express their views on ACI and their understanding of its health knowledge.	
(2) Ask the usual way to understand ACI and help patients distinguish the true and false online information, so as to avoid network fraud.	
(3) Health education: use picture books of ACI knowledge with pictures and pictures to explain the knowledge of ACI symptoms to patients, including the inducing factors of ACI, the inevitability of disease recurrence and impaired limb function after ACI, and the methods of limb rehabilitation training.	
(4) Use stories or metaphors to help patients understand that ideas are ideas, the status quo is the status quo, and ideas cannot exist without the context of the status quo.	
Objective: after the first psychological nursing, patients can correctly understand the disease, to help patients pull open the distance between the ideas and status quo.	

No. 2	Into your life, accept status quo
Basis: ACT—acceptance	
Location: experimental ward (warm, safe and private environment); time: after the basic treatment in the afternoon, before dinner; equipment: wireless audio.	
(1) Encourage patients to express ideas: encourage patients to describe their own worries or fears after the occurrence of the disease thoughts, inner feelings, such as disease treatment, work, life, intimate relationship, and other aspects.	
(2) Negative thoughts normalization: tell patients in the face of the disease, negative emotions is a normal reaction, is the psychological defense instinct, and dos not resist, so as to reduce some unnecessary negative emotions and psychological burden and avoid thinking in the exhaustive.	
(3) Positive thoughts: encourage patients to share the measures taken to deal with the above thoughts or feelings and the effect and praise the positive behavior.	
(4) Accept the status quo: let the patient close his eyes, take a deep breath, and choose a comfortable and relaxed posture to lie or sit well and guide. Allow them to comprehend that inner suffering is common and that we all experience bad feelings when confronted with such issues. Only by embracing the existing quo can you improve yourself by feeling pleased and calm rather than suffering.	
(5) Let patients say to themselves: because I have to face the disease seriously, so I am anxious; I could not sleep because I was trying to figure out how to live my life. Because I realize how important health is, I cannot get depressed.	
Objective: after the second psychological care, patients learn to accept the status quo and remain open to the inner experience they previously avoided.	

No. 3	Observe the self, understand the self
Basis: ACT—self-as-context	
Location: experimental ward; time: after basic treatment in the morning; equipment: white paper, pencil, paper, and glue.	
(1) Self-portrait: let the patient draw a self-portrait of himself on the paper, a simple outline can be.	
(2) Write labels: write their own or others' views on their own, their eating habits, living habits, mentality, personality, occupation, etc., the more complete the better.	
(3) Labeling: ask the patient to stick these labels on their self-portrait.	
(4) Guide the patient to remove the label	
(5) Let the patient tear the label when retelling: this is not me, other people's view is only other people's view; this is not me, I just occasionally have anxiety, need to change; this is not me. Depression is not good for recovery and needs to change. This is not me, I believe I can change bad habits, I am changing. This is not me, the disease is just accidental, not inevitable, I will change.	
Objective: after the third psychological nursing, patients learn to observe themselves and understand themselves. Let patients realize that “I am who I am”	

No. 4	Flexible attention to the now
Basis: ACT—flexible attention to the now	
Location: experimental ward; time: after the basic treatment in the afternoon, before dinner; equipment: wireless audio	
(1) Guide patients to perceive the present: mobilize the five senses, namely, touch, hearing, smell, vision, and taste. First deep breath smooth mood, guide the patient gently close your eyes and experience the feeling of body contact with the bed/floor/seat, experience the temperature of the room, listen to the voices around, trying to explore in the environment, slowly open your eyes, can be seen inside view of the color, and touch the objects around, hand experience and items, the sense of touch.	
(2) Encourage the patient to describe the current feelings: guide the patient to describe in as much detail as possible.	
(3) Be aware of other guides of the present moment: every morning, tell yourself, “I see the light, the darkness will pass, and I will be better.” Every time you eat, tell yourself, “I am replacing nutrition in order to recover quickly.” Every day when receiving infusion therapy, tell yourself, “I will actively work with the medical staff, we will fight the sickness together, I have the courage, and I will be better.” Every time I take a test, I tell myself not to worry; if it's good to find the problem, please assist me in finding the hidden trouble; tell yourself this every day before going to bed: I should rest, rest is to raise enough spirit, believe that tomorrow will be better.	
Objective: after the 4th psychological care, patients can be aware of the present and strengthen the positive belief.	

No. 5	Clarify values, clarify direction
Basis: ACT—valuing	
Location: experimental ward; time: after the basic treatment in the afternoon, before dinner; equipment: white paper, pencil, and paper basket.	
(1) Clarification value	
(2) Help patients to clarify their self-worth: help patients to clarify what is the most important value at present.	
If your life were a book or a TV show, what would you want the ending to be? According to the patient's answer, guide the patient's positive value direction.	
Objective: after the fifth psychological nursing, patients clear self-worth direction, and have a positive attitude to face the status quo.	

No. 6	Set goals, commit to action
Basis: ACT—committed action	
Location: experimental ward; time: after the basic treatment in the afternoon, before dinner; equipment: white paper and pencil.	
(1) Goal setting: to help patients develop specific goals based on value orientation, so that patients are in the leading position in the development of specific plans. Help patients to select suitable and difficult goals for their current situation.	
(2) Commitment to action: in the training or in the realization of the goal, there may be setbacks, once again triggered negative emotions, and actively guide the patient. Objective: after the 6th psychological care, patients make goals in line with their current situation, and commit to action	

No. 7	Relax and sleep peacefully
Basis: ACT—mindfulness and acceptance	
Location: experimental ward; time: after dinner; equipment: wireless audio.	
(1) To guide patients with abdominal breathing: use music with guidance language to focus patients' attention on breathing and every part of the body, relax the body, and avoid entering complex inner activities again. Guide words (speaking slowly): choose a comfortable lying position, preferably a supine position, close your eyes, take a deep breath, put your hands on your abdomen, feel the breath, breath and breath.	
(2) Let the patient be familiar with the music and guide language to relax the body: slowly speak each part of the patient's body, let the patient be familiar with the guide language, to avoid the patient cannot keep up with the guide language and anxious. Let patients relax their body and mind and sleep peacefully.	
(3) Recommend some hypnotic guidance to patients Objective: after the 7th psychological nursing, patients learn relaxation techniques.	

**Table 5:** Comparison of scales after 1 month of psychological nursing.

Item	Scores (min-max)		*Z*	*P* value
	Observation group	Control group		
SAS	51.00 (45-58)	58.00 (52-61)	-8.041	0.001
SDS	53.00 (45-60)	59.00 (54-63)	-8.042	0.001
PSQI	7.00 (4-11)	9 (4-13)	-4.331	0.001
AIS	3.00 (1-6)	6.50 (4-11)	-8.221	0.001
AAQ-II	20.00 (17-24)	31.00 (19-39)	-8.403	0.001
CFQ	22.00 (17-29)	40.00 (20-51)	-8.367	0.001

## Data Availability

All data included in this study are available upon request by contacting with the corresponding authors.
